RETRACTED

# Network Sentiment Analysis of College Students in Different Epidemic Stages Based on Text Clustering

**DOI:** 10.1155/2022/8471976

**Published:** 2022-09-27

**Authors:** Zhenghuai Song, Shanshan Dong

**Affiliations:** ^1^School of Marxism, Yangtze University, Jingzhou, 433020 Hubei, China; ^2^Honghu Market Supervision Administration, Jingzhou, 433020 Hubei, China; ^3^Shanghai Lida University, 201609 Shanghai, China

## Abstract

In order to analyze the evolution trend of public opinion in emergencies and explore its evolution law, this paper constructs a network sentiment analysis model based on text clustering, where the emotion analysis part is based on the pretraining BERT model and BiGRU model, in which BERT is used as the word embedding model to extract the feature vector of emotional text and BiGRU is used to extract the context of the text feature vector to accurately identify the sentiment polarity of public opinion data. In addition, the *K*-means clustering algorithm and Kolmogorov-Smirnov *Z* test were used to divide the different epidemic stages. Compared with other methods, the model proposed in this paper has a great degree of improvement in accuracy, recall, and *F*1 score index, which provides an opportunity reference and effective detection means for schools at all levels to carry out timely mental health education and psychological intervention for students.

## 1. Introduction

At the beginning of the new year 2020, Wuhan began to have pneumonia of unknown origin, and the COVID-19 pandemic began to spread to the whole country. Since the outbreak of the epidemic, in order to effectively prevent the spread of pneumonia, home isolation policy has been implemented in many places. Therefore, during the period of the epidemic, the research on emotion adopts the form of network questionnaire based on self-report method to measure emotion. Although the form of online questionnaire is more convenient for the subjects, due to the limited sample size, Hawthorne effect, and social approval, the validity of emotional measurement results is affected to a certain extent [1].

Network emotion is a kind of social emotion, which is the most direct and real reflection of the current social emotion. It has three characteristics: low tipping point, abnormal emotion, and obvious political direction. Bi et al. [2] believed that in the Internet environment, social emotions can be more easily expressed through the network. Under the trigger of network events, the collective emotional reaction of netizens forms the network emotion. Dong et al. thought that the wider spread of real emotions through Internet technology is network emotion [3]. It is worth noting that due to its convenience and high coverage, the Internet has become an important platform for people to exchange and discuss and express their opinions in this special period. Network text has become an important carrier for people to vent their emotions, which contains rich emotional information. Due to the anonymity of the network, the emotional information contained in the network text is more authentic [4]. Therefore, the network text has become a valuable research data for emotion research during the epidemic period. Using network text to study emotion, understanding the characteristics and change trend of network emotion can be more timely and accurate to understand the emotional status of students during the epidemic, identify the changes and characteristics of emotions, which helps colleges and universities to grasp the mental health status of students, and timely strengthen the mental health education of students and has important practical significance for government departments to understand and respond to emergency network public opinion.

RETRACTED

Therefore, this paper constructs a network sentiment analysis model based on text clustering. Combined with *K*-means clustering algorithm and Kolmogorov-Smirnov *Z* test, the different epidemic stages were divided, and the network emotion of college students in different epidemic stages was analyzed by word frequency extraction results and emotional value calculation.

## 2. Related Work

### 2.1. User Emotion Classification

As the most direct embodiment of network social mentality and social emotion, grasping the state and change of current network emotion is helpful to understand the change of current social mentality. Therefore, it is very important to analyze the behavior of users affected by epidemic situation. Li et al. [5] analyzed the microblog data and found that after the outbreak of the epidemic. On the whole, the public have more negative emotions, pay more attention to the health of themselves and their families, and ignore the leisure and entertainment, friends' feelings, and other things [5]. Chen [6] made a comparative analysis of microblog and Twitter and found that users form these platforms tend to publish more content when the number of confirmed cases increases. The author also analyzed the main epidemic events that led to anger, disgust, fear, happiness, sadness, surprise, and other emotions. In addition to the above research on the characteristics of the blog itself, there are also some work focused on the transmission characteristics of epidemic related content. Zhang et al. proposed seven types of information needs related to people's livelihood, including epidemic prevention suggestions, government measures, donations, emotional support, seeking help, questioning and monitoring, and refuting rumors [7], and analyzed the characteristics of emotion, hashtag, and publisher information of each type of information needs, which provided help for decision-makers to find and solve livelihood problems. Gao et al. found that mental problems such as depression and anxiety disorder caused by the COVID-19 pandemic were associated with frequent acceptance of information on social media. During the epidemic period, the public tend to use search engines to obtain the news, disease, treatment, and other information related to the epidemic, and the analysis of search engines can better understand the public's concerns, information needs, and other behaviors [8].

RETRACTED

### 2.2. Network Sentiment Analysis Model

Many scholars have devoted themselves to the construction of network emotion recognition and analysis model. In the study of lexicographic sentiment analysis based on the “emotion dictionary + rule” mode, Hamouda and Akaichi established an emotional vocabulary library containing emoticons for emotion recognition [9], and Gaikwad and Joshi proposed that different emotional words and symbols should be given different weight values to distinguish their contribution to the emotional polarity of the text [10]. However, the method based on emotion dictionary has its limitations; that is, the emotion of a text is not accumulated by the emotional polarity of its constituent words. Support vector machine (SVM) and naive Bayes algorithm (NB) are often used for sentiment classification in network sentiment analysis based on machine learning. Sharma and Dey established an integrated text sentiment classifier by combining the classification performance of boosting and SVM as a basic classifier, and the research results show that the accuracy of the integrated sentiment classifier is significantly higher than that of a single SVM classifier [11]. Perikos and Hatzilygeroudis combined Bayesian classifier and maximum entropy classifier to establish another integrated classifier, which can conduct in-depth analysis of natural language sentences and has high accuracy of emotion classification [12]. Tripathy et al. divided the text according to the combination of basic word units and used naive Bayes, maximum entropy, support vector machine, and random gradient descent method and combination method to conduct emotional analysis of online reviews and compared the differences and advantages of each method [13].

Emotion analysis based on deep learning can improve the accuracy of text classification [14], where CNN and RNN are often used as modeling tools for emotion analysis. Zhou et al. proposed the LSTM (Long Short-Term Memory Network) model based on multiattention mechanism and analyzed the network emotion of netizens in the event of “Huawei P10 flash” [15]. Hu et al. established a keyword thesaurus based on the LSTM model to mine potential languages in texts, which further improved the accuracy of text sentiment polarity analysis [16]. Ma et al. established a perceptual LSTM model, where a superimposed attention mechanism composed of statement level and target level attention models were added to LSTM [17].

RETRACTED

### 2.3. Public Opinion Evolution Analysis

The evolution process of public opinion events often has a life cycle. The researchers have explored the process of public opinion communication. These studies divide public opinion into stages according to the sequence of events and the life cycle of development according to different angles and build models. Zhang et al. believe that the public opinion of COVID-19 epidemic shows periodic changes; the network model based on evolutionary chain has a significant community structure in geospace, which can be divided into seven regions [18]; Tan et al. divided the development process of online public opinion into four stages: incubation, diffusion, transformation, and attenuation [19]. Lian et al. simplified the evolution process into three stages: initial propagation, rapid diffusion, and extinction [20]. At the same time, scholars have also analyzed the characteristics of each stage of the network public opinion. However, different emotion analysis methods lack a unified accuracy index, and in the emotion analysis based on machine learning, the accuracy of the model is low, while the ecological validity of the network emotion analysis model for a certain event is poor, which is difficult to apply to the analysis of network emotion under other events.

## 3. Network Sentiment Analysis Model Based on Text Clustering

### 3.1. Framework of Emotional Analysis

A comprehensive analysis framework “attention—emotional polarity” of COVID-19 pandemic was constructed, as shown in Figure 1. Attention refers to the number of texts contained in each topic according to the document topic matrix, which can reflect the students' attention to each topic of the epidemic. Emotional polarity refers to the average emotional score of the literature contained in each topic, which can reflect the user's emotional attitude towards the various themes of the epidemic.

### 3.2. Text Sentiment Analysis

After the COVID-19 incident broke out, netizens basically had a large number of emotional words or could judge their emotional attitude, such as “uncomfortable,” “very sad,” “better,” and “strong,” which directly reflected the psychological and emotional trend of netizens at that time. Sentimental analysis is an important technology of sentiment recognition and opinion mining in the field of natural language processing, which is also an important part of public opinion analysis. Based on the above emotional words, this paper proposes the trend of netizens' attitudes towards hot events, which are mainly divided into “positive” and “negative” emotions. The main process of text sentiment analysis is as follows:

1. Firstly, the original text is preprocessed, including custom dictionary, stop dictionary, and noise removal
2. Then, the training set is divided into training set and test set
3. Finally, the corpus is extracted from the training set for emotional retrieval, classification, and extraction of opinion words. The specific steps are shown in Figure 2

RETRACTED

### 3.3. *K*-Means Clustering

The object-attribute structure describes the specific attributes of a specific object. Each object has one or many attributes. Assuming that an object has *m* attributes, this data structure can be converted into an *n* × *m* matrix as follows:

(1) $$\begin{array}{c} \left[\begin{array}{cccc} x_{11} & x_{12} & \cdots & x_{1m}\\ \cdots & \cdots & \cdots & \cdots \\ \cdots & \cdots & \cdots & \cdots \\ x_{n1} & x_{n2} & \cdots & x_{nm} \end{array}\right]. \end{array}$$

The object-object structure quantifies the differences between objects by the distance *d*(*i*, *j*). The closer *d*(*i*, *j*) gets to 0, the more similar *i* and *j* are, so they can be classified into one class. On the contrary, the larger the value is, the more different the object is. Thus, it can be obtained that its matrix is a diagonal matrix as follows:

(2) 0    d2,10   d3,1d3,20  ⋯⋯⋯⋯ dn,1dn,2⋯⋯0.

The time complexity of *K*-means clustering algorithm is lower than other algorithms, and it can also achieve better clustering effect. Moreover, the *K*-means algorithm is easy to implement and has fast clustering speed. So *K*-means algorithm is selected to cluster text. The idea of *K*-means clustering algorithm is to calculate the center point continuously and divide it circularly until the final clustering is unchanged. The clustering process is shown in Figure 3.

1. Determine the types of sample points to be clustered *k*
2. Select *K* points as initial centers *C* = {*c*_1_, *c*_2_, ⋯, *c*_*k*_}
3. Calculate the distance between sample point *x*_*i*_ and the initial center, and divide categories according to the distance
4. Recalculate the new cluster centers by using

(3) $$\begin{array}{c} c_{i}=\frac{1}{\left|c_{i}\right|}\Sigma_{x\in c_{i}}x, \end{array}$$

where *c*_*i*_ is the distance from each cluster to the cluster center

(5) Calculate and optimize the loss function by using

(4) $$\begin{array}{c} J\left(c^{\left(1\right)},c^{\left(2\right)},\cdots ,c^{\left(m\right)};\mu_{1},\mu_{2},\cdots ,\mu_{k}\right)=\frac{1}{m}\overset{m}{\underset{i=1}{\sum }}\;{||x^{\left(\text{i}\right)}-\mu_{c}\left(i\right)||}^{2}, \end{array}$$

where *μ*_*c*_(*i*) represents the nearest clustering center to *x*^(i)^. *x*_*i*_ represents the sample point. The essence of *K*-means is to move the center point and make it gradually close to the data “center,” that is, to minimize the objective function, which is the sum of squared distances between each point and its cluster centroid

RETRACTED

### 3.4. Sentiment Analysis Model

In order to analyze the sentiment polarity and evolution of public opinion better, as shown in Figure 4, this paper proposes an emotional polarity analysis algorithm based on emotional features to identify the sentiment of public opinion data during the epidemic period. A layer of BiGRU is added after the BERT model to better capture the context relationship between word vectors, and the data of public opinion during the epidemic period were accurately identified by emotion polarity, and the hot spots of public opinion under different emotional polarity were explored by calculating word frequency.

The traditional word vector model is suitable for analyzing short sentences and simple sentences. In order to solve the problem of polysemy, we should also consider the relationship between text and word. Compared with traditional text sentiment analysis, BERT model can better cover the relationship between contexts.

The text features are extracted by the BERT base. For the input text, BERT can be used for feature extraction by using

(5) $$\begin{array}{c} C_{n}=\text{BERT}\left(tn\right). \end{array}$$

The model takes the output *C* of the [CLS] marker at the last layer of BERT training and adds the weight *W* as the input of the bidirectional GRU model, i.e.,

(6) $$\begin{array}{c} a_{i}=g\left(W_{a}\times c_{i}+b\right), \end{array}$$

where 1 ≤ *i* ≤ *n*, *n* is the characteristic dimension of BERT output; *b* is the offset; a function *g* is the Sigmoid function.

The model feeds the input vector into BiGRU, uses two GRUs to calculate the vector sequence from different directions, and finally combines the results of the two directions for output, namely,

(7) $$\begin{array}{c} h_{i}=\text{BiGRU }\left(a_{i}\right). \end{array}$$

Then, the softmax function is used to classify the feature vectors output by BiGRU, and the final identification result of emotional polarity is obtained.

## 4. Model Validity Analysis

### 4.1. Data Acquisition

This paper uses the Scrapy crawler framework to crawl and analyze the mobile site <http://s.weibo.com>. Because the public opinion texts during the epidemic period first changed from “viral pneumonia” to “COVID-19 pandemic in 2019,” the official names were defined as “2019 nCoV” and “COVID-19” in the midterm. In order to crawl the integrity of the data, using “2019 nCoV,” “COVID-19,” “pneumonia,” and “epidemic situation” as keywords, a large number of microblog data from January 2021 to August 2021 were crawled. The training set is used to train the public opinion sentiment polarity model during the epidemic period, and the verification set is used to verify the effectiveness of the proposed method.

RETRACTED

### 4.2. Experimental Parameters

The loss function used in this paper is cross-entropy loss function, and Adam algorithm is used to optimize the loss function. The learning rate, batch size, iteration times, and maximum text length are set to 1*e* − 5, 16, 2, and 140, respectively. In order to verify the effectiveness of the proposed method, the experimental results are compared with those of several mainstream experimental methods (TF-IDF+LR, LSTM, TextCNN, and BERT-Base). In addition, the accuracy, recall, and *F*1 score were used to evaluate the experimental results. Among them, recall is the number of correct judgments for a class divided by the number of classes in the test set.

### 4.3. Results and Analysis

The performance of different experimental methods is shown in Table 1.

As can be seen from Table 1, compared with other methods in the analysis of public opinion emotion during the epidemic period, the accuracy rate, recall rate, and *F*1 score of this method are 0.753, 0.714, and 0.716, respectively. Compared with the TF-IDF+LR model with the worst training effect, the three indexes are increased by 23.8%, 18.8%, and 19.5%, respectively. This may be because in terms of large-scale data, the BERT pretraining model obtained by training can cover more information to deal with the public opinion data during the outbreak. In addition, after the introduction of BiGRU, the proposed method can extract the relationship between words in public opinion data more effectively.

## 5. Analysis of College Students' Network Emotion in Different Epidemic Stages

### 5.1. Classification of Epidemic Stages

Because the sample feature vectors used in each project are different, we can choose to measure the numerical distance or the directional correlation according to the distribution characteristics of the selected feature vectors and the project requirements. The optimal number of topics *K* is determined by four indicators: cosine distance, KL difference distance, logarithmic likelihood, and JS distance, namely, Cao Juan 2009, Arun 2010, Griffiths 2004, and Deveaud 2014 [21]. The results are shown in Figure 5. With the increase of the number of topics, the three reference values of Cao Juan 2009, Arun 2010, and Deveaud 2014 fluctuated and decreased, while Griffiths 2004 showed a fluctuating increase. With the number of topics increasing, the computational cost of the model increases correspondingly, and the overfitting phenomenon is easy to appear. However, when the number of topics is 4, there is a local optimal value. If the number of topics continues to increase, the profit is less than the investment. Therefore, the optimal number of topics is determined to be 4 based on the four indicators.

RETRACTED

The specific topic content of each cluster is as follows.

Cluster 1: it mainly describes the psychological and emotional changes of students, reflecting that students pay more attention to the way of learning in school.

Cluster 2: it mainly describes the students' fear of the outbreak of the epidemic and their dissatisfaction and complaint about the long-term isolation at home.

Cluster 3: it mainly describes the notice of the beginning of school and the students' desire and expectation for the coming school life.

Cluster 4: it mainly describes that the students have adapted to the measures of epidemic prevention and control and shifted their attention from the epidemic situation, home isolation, and online class to the coming school day.

According to the calculation results of emotional mean value in Figure 6, there are two lowest peak points and one peak point in the epidemic situation. The low peak point is near February 26 and April 30, respectively, and the peak point is near August 31. The lowest emotional value is only 0.3, and the highest emotional value is more than 0.8. Before April 6, the emotional value fluctuated greatly, maintained between 0.3 and 0.5, and rose steadily after April 30. The overall emotional value was maintained above 0.6. Taking February 1, February 27, April 7, and August 31 as the starting dates of the initial period, outbreak period, recovery period, and growth period, the Kolmogorov-Smirnov *Z* test was conducted. The results are shown in Table 2.

From the results, it can be found that there is a significant difference between the recovery stage and the growth stage (*P* < 0.01), where the average emotional value has a significant increase; in addition, there was no significant difference between the initial stage and the recovery stage (*P* = 0.9858). Therefore, according to the difference of network emotion distribution, the students' network emotion stage during the epidemic period was divided into the following four stages: initial period (February 1 to February 26), outbreak period (February 27 to April 6), recovery period (April 7 to April 30), and growth period (May 1 to September 1).

RETRACTED

### 5.2. Analysis of College Students' Network Emotion in Different Stages

After determining the time division of the emotional stage of college students during the epidemic, descriptive statistics were made on the amount of microblog releases at different stages and the emotional values calculated by the model, as shown in Table 3.

#### 5.2.1. Initial Period

In the initial stage, the positive emotion microblog accounted for 59.3%, and the emotional value was 0.645 ± 0.396. The overall potency of online emotion was positive. In this stage, the COVID-19 pandemic is in an explosive growth period. In order to effectively prevent the further spread of the epidemic, local governments have implemented home isolation measures. The student group has not yet had a clear understanding of the impact of the epidemic on their own health, and this period is also the winter vacation period when most schools have not yet returned to school. Therefore, the number of microblogs related to the start of school is relatively small (*N* = 1387). The result of word frequency extraction in the initial period is shown in Figure 7, in which, the frequency of the word “Holiday” (204 times) was higher than that of “Epidemic” (188); “Operation” (142 times) ranked fourth; in addition, “When” (75 times) was 13th. Although the word “Online class” (69 times) also appeared in the 16th place of word frequency statistics, the frequency was less.

It can be seen that at the initial stage, students have not fully understood the delay of school after the epidemic, more attention is focused on holidays and homework, and less attention is paid to the online class as an alternative form of face-to-face class. During this period, besides the epidemic itself, more of the stimuli that affected the students' collective emotions were their own studies and the unknown arrangements for the school's return to classes.

#### 5.2.2. Outbreak Period

During the outbreak period, the positive emotion microblog accounted for 49.8%, and the emotional value was 0.559 ± 0.414. The overall potency of online emotion was negative. During this period, the local education departments and colleges and universities have issued the notice of continuing to delay the opening of school, which also means that the students' time of isolation at home and online classes continues to be extended, and no clear opening data has been released. The number of microblog release in the outbreak stage was the largest (*N* = 34615), and the overall emotional distribution of the students in this stage decreased significantly compared with the initial stage (*P* = 0.000), and there were significant differences between the distribution of the emotional values in the other two stages. The extraction results of word frequency in the outbreak period are shown in Figure 8.

RETRACTED

The frequency of words such as “School” (6980 times), “At home” (4900 times), and “Online class” (3521 times) during the outbreak period was similar to that of the whole word frequency statistics. In addition, we can find that the words “Hurry” (1737 times) and “Hope” (1686 times) appear in the 17th and 18th places of the word frequency statistical results. From the above results, it can be seen that the overall mood of students in the outbreak period is more negative than that in the initial stage. The reason for this situation may be due to the dissatisfaction and complaint about the long-term isolation at home, and online classes also make students feel more negative experience than normal in-school classes.

#### 5.2.3. Recovery Period

During the recovery period, the positive emotion microblog accounted for 59.5%, and the emotional value was 0.649 ± 0.394. The overall potency of online emotion was positive. There was a significant increase in the distribution of emotional values in the recovery period compared with the outbreak period (*P* = 0.000), where the students showed more positive emotions in general. However, there was no significant difference between the distribution of emotional value in this stage and that in the initial stage (*P* = 0.926), so the overall emotion in this stage returned to the state before the outbreak period.

The results of word frequency extraction in the recovery period are as shown in Figure 9, “Finally” (613 times) and “First day” (587 words) are in the 9th and 12th places, respectively. At the same time, it should also be noted that “Unwilling” (1032 times) and “Examination” (749 times) appear in the fifth and eighth places of the statistical results, which indicates that in the recovery period, the academic pressure is also an important source of negative emotions in the overall emotional composition. In addition, the word “Epidemic” did not appear in the high-frequency words, indicating that in this stage, the epidemic situation has no longer become an important factor affecting the overall mood of students.

#### 5.2.4. Growth Period

The results of word frequency extraction in the growth period are as shown in Figure 10. During the growth period, the positive emotion microblog accounted for 64.5%, and the emotional value was 0.688 ± 0.386. The overall potency of online emotion was positive. According to the results of emotional value distribution, the emotional value of the growth stage was significantly higher than that of the recovery stage (*P* = 0.000), and there were significant differences between the emotional value distribution and the other three stages. At this stage, the overall emotion of students is the most active stage in all stages.

RETRACTED

According to the results of word frequency ranking, the words “Tomorrow” (1472 times), “Today” (1436 times), and “Time” (1328 times) related to time accounted for the second, third, and fifth places, respectively; “Finally” (1177 times), “ha ha ha” (1135 times), “Happy” (833 times), “Hope” (825 times), and “Come on” (734 times) are the 6th, 7th, 13th, 14th, and 20th places, respectively. The beginning of school and the coming of school have become the important reasons to promote the overall positive trend of students' emotions. The same as the recovery period, “Epidemic” did not appear in the statistical results; in addition, “Online class” and “At home” did not appear in the statistical results for the first time, which shows that the epidemic situation has been fully controlled in the growth period, where students have shifted their attention from the epidemic, home isolation, and online classes to the coming day of school.

To sum up, the negative emotions of students during the epidemic period mainly come from the epidemic itself, the measures of preventing epidemic at home, the academic burden brought by home-based learning with online courses, and the unknown of the beginning of school. But after the growth period, the overall network emotion began to show a positive state, and with the change of time, the emotional valence showed an upward trend.

## 6. Conclusion and Suggestion

### 6.1. Conclusion

In this paper, a sentiment polarity analysis algorithm based on sentiment features is proposed to identify the sentiment of public opinion data during the epidemic. A BiGRU layer is added to the BERT model to better capture the contextual connections between word vectors. This paper constructs a network sentiment analysis model based on text clustering, where the *K*-means clustering algorithm and the Kolmogorov-Smirnov *Z* test were used to classify different epidemic stages, and the word frequency extraction results and emotional value calculation were used to analyze the online emotions of college students in different epidemic stages. The experimental results show that the accuracy, recall, and *F*1 score of the proposed model are greatly improved compared with other methods. During the epidemic period, the students' network emotion stage can be divided into four stages: the initial stage, outbreak stage, recovery period, and growth stage. The negative emotions of students during the epidemic period mainly come from the epidemic itself, the measures of preventing epidemic at home, the academic burden brought by home-based learning with online courses, and the unknown of the beginning of school. But after the growth period, the overall network emotion began to show a positive state, and with the change of time, the emotional valence showed an upward trend.

RETRACTED

### 6.2. Suggestions

Based on the above analysis, the following suggestions can be put forward for the psychological construction of college students during the epidemic period:

1. During regular prevention and control of the COVID-19 pandemic, during a sudden outbreak, schools and local education departments to ensure the related policy and the school to arrange timely release, let the students know the arrangements to school first, in order to prevent the outbursts in network within the period due to the negative emotions produced and spread of unknown cause
2. In the recovery and growth stages of network emotion, attention should be paid to strengthen students' awareness of self-protection, continue to implement the epidemic prevention work, to prevent the emergence and spread of local epidemics due to slack and negligence

## Figures and Tables

**Figure 1:** Framework of emotional analysis.

**Figure 2:** Process of text sentiment analysis.

**Figure 3:** *K*-means clustering process.

**Figure 4:** Framework of sentiment analysis model.

**Figure 5:** Cluster analysis results.

**Figure 6:** Calculation results of emotion value.

**Figure 7:** Extraction results of word frequency in the initial period.

**Figure 8:** Extraction results of word frequency in the outbreak period.

**Figure 9:** Extraction results of word frequency in the recovery period.

**Figure 10:** Extraction results of word frequency in the growth period.

**Table 1:** Performance of different experimental methods.

Method	Accuracy	Recall	*F*1 score
TF-IDF+LR	0.608	0.601	0.599
LSTM	0.652	0.638	0.640
TextCNN	0.641	0.633	0.631
BERT-Base	0.749	0.709	0.713
Proposed model	0.753	0.714	0.716

**Table 2:** Kolmogorov-Smirnov test of epidemic stages.

	1	2	3	4
Initial period	—			
Outbreak period	3.708^∗∗∗^	—		
Recovery period	0.547	9.858^∗∗∗^	—	
Growth period	2.492^∗∗∗^	17.631^∗∗∗^	5.448^∗∗∗^	—

Note: ^∗∗^*P* < 0.001.

**Table 3:** Analysis of college students' network emotion in different stages.

Stage	Total microblog releases	Positive emotion microblog release	Proportion (%)	Emotional value
Initial period	1387	822	59.3	0.645 ± 0.396
Outbreak period	34615	17239	49.8	0.559 ± 0.414
Recovery period	13721	8162	59.5	0.649 ± 0.394
Growth period	22273	14357	64.5	0.688 ± 0.386

RETRACTED

## Data Availability

The data that support the findings of this study are available from the corresponding author upon reasonable request.
